The article "Sevoflurane Inhibits lncRNA HOTAIR-Modulated Stability of HK2 mRNA in a m6A-Dependent Manner to Dampen Aerobic Glycolysis and Proliferation in Lung Cancer" was retracted in 2023. Reasons: signs of a paper mill; compromised peer review; unreliable results or conclusions.

# Sevoflurane Inhibits lncRNA HOTAIR-Modulated Stability of HK2 mRNA in a m6A-Dependent Manner to Dampen Aerobic Glycolysis and Proliferation in Lung Cancer

**DOI:** 10.1155/2022/4668774

**Published:** 2022-07-06

**Authors:** Xuefeng Sun, Qiyong Li, Ling Yang

**Affiliations:** ^1^Department of Anesthesiology, The Second People's Hospital of Three Gorges University (Yichang Second People's Hospital), Yichang, 443000 Hubei Province, China; ^2^Radiology Department, The Second People's Hospital of Three Gorges University (Yichang Second People's Hospital), Yichang, 443000 Hubei Province, China; ^3^Hemodialysis Room, The Second People's Hospital of Three Gorges University (Yichang Second People's Hospital), Yichang, 443000 Hubei Province, China

## Abstract

Previous studies have shown that sevoflurane has an inhibitory effect on tumor cells. So far, the effect of sevoflurane on hepatocellular carcinoma needs to be confirmed by more studies. HOX transcript antisense intergenic RNA (HOTAIR), a long noncoding RNA (lncRNA), has been shown to enhance cancer cell proliferation and medication resistance. The inherent importance and biological function of HOTAIR in the course of lung cancer (LC) is, however, poorly unclear. HOTAIR was shown to be highly elevated in LC cells in this investigation. Impairment of function trials with sevoflurane indicated that it has anticancer effects on LC cell growth, apoptosis, and aerobic glycolysis. In a mechanistic manner, HOTAIR was related to HK2 mRNA and promoted expression and constancy. Additional research revealed that HOTAIR coupled with hexokinase 2 (HK2) mRNA and favorably controlled its stabilization in a traditional-component way. By HK2, the LC enhancement role was mediated. In summary, our data show that HOTAIR promotes the synthesis and proliferation of LC glycogen by increasing the transcription of HK2, and HOTAIR is likely to be a potential treatment for LC patients.

## 1. Introduction

Lung cancer (LC) is one of the deadliest cancers, except for a marginal improved life throughout the last thirty years [1]. Moreover, chemotherapy is the main treatment for advanced or metastatic lung cancer, but because of the intrinsic or acquired resistance to chemotherapy, many patients eventually develop antichemotherapy. As a result, elucidating the biological pathways causing chemotherapeutic tolerance could lead to the identification of promising agents for LC therapies.

Prior research suggests that sevoflurane could stimulate tumor cellular activities and dissemination. However, more evidence suggests that sevoflurane inhibits cancerous cellular growth. So far, the effect of sevoflurane on hepatocellular carcinoma has not been determined. Nevertheless, whether high-intensity focused ultrasound (HIFU) has an effect on the invasion and metastasis of lung cancer remains unclear.

Long noncoding RNAs (lncRNAs) are a new type of RNAs those are longer than 200 tandem repeats but lack effective protein-coding potential [2]. A couple of lncRNAs that engage in the hematological regulation system have previously been explored [3]. Indeed, it has been proposed that certain lncRNAs may operate as target repressed genes or tumorigenesis since they affect the transcription of genes encoding in tumorigenesis and development, along with tolerance to medication, actively or passively [4]. Taken an example, antisense RNA3 of homeobox protein B8 gene (HOXB-AS3) modulates ribosome translation in NPM1-mutated leukemias [5]. Myocardial infarction-associated transcript (MIAT) also hastens the course of acute myeloid leukemia by adversely regulating miR-495 [6]. GAS5 modulates carcinogenesis and dissemination in human B myeloid leukemia by syphoning miR-222 [7]. HOX transcript antisense intergenic RNA (HOTAIR) is a human gene located between homeobox (HOX) C11 and HOXC12 on chromosome 12. It is the first example of an RNA expressed on one chromosome that has been found to influence transcription of HOXD cluster posterior genes located on chromosome 2. HOTAIR is highly expressed in metastatic breast cancers. High levels of expression in primary breast tumors are a significant predictor of subsequent metastasis and death. HOTAIR is able to promote myeloma cellular proliferation and drug endurance. HOTAIR potentially promotes cellular proliferation and treatment failure by activating the p38-JNK-MAPK networks [8]. The inherent relevance and essential part of HOTAIR in the development of LC, but at the other hand, is mainly unclear. Within aerobic environment, malignant cells take up glycogen and convert it to lactic, which itself is recognized also as the Warburg impact [9]. Enough nucleotide, polypeptide, and lipid generated from such a form of gluconeogenesis are necessary for carcinoma cell fast development and differentiation [9]. The Warburg effect is activated by upregulating or downregulating the presence of different percentage kinases [10]. Targeting Warburg effects have become an important part of antitumor treatments; for instance, in JAK2V617F-positive hematopoietic stem cell malignant tumors, hypoxia-inducible factor 1 (HIF-1) brings a new clinical application [11]. The pathways behind the beginning and maintenance of the Warburg effect activities in LC, nevertheless, are unknown.

Another pathway of HOTAIR in regulating the development of LC may be the Nmurine 6-methyl adenosine (m6A) pathway, which is the regulation of NMel 6 adenine nucleotides in mRNA. In human cells, m6A change is the most common messenger RNA change, with the highest frequency in the string [12]. Compared with other mRNA changes, m6A modification is dynamically reversible and, like DNA and epigenetic variation, regulates the maturation, translation, and destruction of precursor mRNA [13]. Methyltransferases (METTL3, METTL14, and WTAP) and demethylases (FTO and ALKBH5) are mainly responsible for m6A changes [13]. During the whole process of intracellular homeostasis and tumorigenesis, changes in m6A have been found to control stem cell differentiation and renewal by affecting the turnover of mRNA. New data show that m6A mutation is associated with the occurrence and development of a variety of human cancers [14]. For example, in leukemia, the addressable RNAm6A sensor YTHDF2 specifically damages malignant cells [15]. METTL14 promotes leukemia through m6A gene modification [16]. At present, the role of m6A in LC is not clear, so this paper will carry out the research on m6A.

In present study, we demonstrated that HOTAIR was greatly upregulated in LC cell lines. HOTAIR's carcinogenic effects on LC cellular growth, apoptosis, and aerobic glycolysis were discovered by loss-of-function assays. HOTAIR binds to hexokinase 2 (HK2) mRNA and promotes its translation and maintenance through a mechanism. Further research revealed that HOTAIR connected to HK2 mRNA and favorably controlled its stabilization in an FTO-dependent way. HOTAIR's LC enhancement effects were mediated by HK2. Our research not only identified HOTAIR as a new target, but also revealed new mechanisms regarding the regulation of glucose utilization and anaerobic glycolysis in LC.

## 2. Materials and Methods

### 2.1. Cell Culture

Human lung cancerous cells (A549 cell lines) were obtained from American Type Culture Collection (ATCC; Manassas, VA, USA). Cells were grown at 37°C in a humid environment of 5% CO_2_ in RPMI-1640 medium (GIBCO, Gaithersburg, MD, USA) containing 10% heat neutralized fetal calf serum (GIBCO, Gaithersburg, MD, USA).

### 2.2. Plasmid Construction and Transfection

The negative control shRNA and HOTAIR shRNA were supplied from Genechem (Shanghai, China). GeneCopoeia provided the pcDNA3.1-HK2 (HK2) and pcDNA3.1-control (vector) constructs (Guangzhou, China). Transfection was carried out by Lipofectamine 3000 (Life Technologies, USA) in accordance with the company's recommendations.

### 2.3. Quantitative Real-Time PCR (qRT-PCR)

Total RNAs were isolated applying TRIzol reagent (Carlsbad, CA, USA) and reversely transcribed into cDNA by Power SYBR® Green PCR Master Mix kit (Applied Biosystems, USA). Q-PCR used DNA Engine Opticon 2 Real-Time Cycler (MJ Research, Inc.). GAPDH was utilized as an internal standard, and the sequences used here qRT-PCR are listed below: HOTAIR, 5′-AGCGAAGTCCCGAACGACGA-3′ (forward) and 5′TGGGCATTTCCAACGGGCCAA-3′ (reverse); GAPDH, 5′ATGATGACATCAAGAAGGTGGTG-3′ (forward) and 5′CCATGAGGTCCACCACCCTGTTG-3′ (reverse); and HK2, 5′CGCGCACAATCCCTACCCATCGCC-3′ (forward) and 5′-CTTCCAGAGGAGAGAGTTGGTTCTG-3′ (reverse).

### 2.4. Cell Proliferation Assay

The cellular growth rates of LC cells were detected using the cell counted kit-8 test kit (Dojindo, Kumamoto, Japan). The cells were planted onto multiwell plates at a density of 2000 cells/well. The plates were then incubated at 37°C with 5% CO_2_. The cells were incubated with CCK-8 liquid (10 ml/well) for 2 hours at the time specified by determination of OD value at 450 nm. All the experiments were copied at least three times.

### 2.5. Apoptosis Assay

Flow cytometry would be used to identify apoptotic cell death using only a cell apoptosis stain kit (Invitrogen). Cells and supernatant were harvested and centrifuged for 5 minutes at 1500 rpm. The cells were then rinsed in PBS and resuspended in lysis buffer before being combined with Annexin V-APC/7-AAD. The cells were placed into flow tubing and incubated in the dark for 20 minutes at room temperature. Flow cytometry was used to examine the specimens (FC500 MPL, Beckman Coulter).

### 2.6. Western Blot Assay

Protein concentrations were determined using BCA Protein Assay kit (Beyotime, Shanghai, China) after the cells were digested in Lysis buffer. SDS-PAGE was used to segregate the cellular extracts, which were then loaded to a PVDF film that had been coated in solution and coated with primary antibodies. Then, the PVDF membranes were then incubated overnight with secondary antibodies and visualized by enhanced chemiluminescence kit (Thermo Scientific, USA). Abcam provided the HK2 and actin antibodies used in this study.

### 2.7. Subcellular Fractionation

According to the PARIS KIT technique (Life Technologies, Carlsbad, CA), the centrifugation was done for 5 minutes to get the nuclei and cytoplasmic components. GAPDH, HOTAIR, and U6 mRNA levels were measured using the qRT-PCR technique.

### 2.8. Glucose Consumption, Lactate Production, and ATP Generation Assay

The filtrates of growth medium and cells were obtained individually for assessing glucose intake and lactic generation in LC cells planted in a 96-well plate. Glucose intake levels were assayed using a Glucose Uptake Assay box (BioVision, Milpitas, CA, USA). The lactate was detected by lactic acid kit II (BioVision). The ATP colorimetry (BioVision) was used to measure ATP creation based on the operator's procedure.

### 2.9. Extracellular Acidification (ECAR) and Oxygen Consumption Rate (OCR)

The ECAR and OCR were measured using the analyzer and kits, respectively. Examinations were carried out in accordance with the company's instructions. Briefly, 2 × 10^4^ cells were planted into the special cell-plate wells. After baseline assessment, for ECAR, glucose, oligomycin (oxidative phosphorylation inhibitor), and 2-DG (glycolytic inhibitor) were orderly injected at shown time points; and at the relevant time frames, oligomycin, the dynamic regulator of *β*-oxidation FCCP, and the cellular complex inhibitor active ingredient were administered, along with the mitochondria complex III antagonist antimycin A (Rote/AA). LC data was assayed by Seahorse software.

### 2.10. RNA Immunoprecipitation (RIP) and Methylated RNA Immunoprecipitation (MeRIP) Assays

RIP and MeRIP assay were performed using RNA Immunoprecipitation (RIP) Kit (Bersin Bio) according to its instruction.

### 2.11. Luciferase Reporter Assay

HK2 promoter region was cloned into pGL3 plasmid. pGL3 or pGL3-HK2 and pRL-TK were transfected into LC cells with HOTAIR knockdown. After two days, the activity was measured using luciferase assay system.

### 2.12. Regimen of Lung Cancer Cells Exposed to Sevoflurane

The cell culture plate is placed in a sterile airtight container with inlet and outlet connectors. The anesthesia machine (GE Healthcare Life Sciences, Chalfont, UK) is connected to the air inlet and to the sevoflurane atomizer (sevoflurane; Abbott, Albert Park, Illinois) to provide sevoflurane gas to the container (mixed with 95% O_2_ and 5% CO_2_). The concentration of sevoflurane in the container is monitored by a gas monitor connected to the outlet of the container (PM8060, Drager, Lubeck, Germany). The cells were treated with sevoflurane for 6 hours, then cultured under normal conditions for 24 hours, and then further analyzed.

### 2.13. Statistical Analysis

LC statistical analyses used GraphPad 9.0 and displayed as mean ± SD. Great differences were confirmed by *T* test or one-way analysis of variance (ANOVA). *P* value < 0.05 was seen as a significant difference.

## 3. Results

### 3.1. HOTAIR Is Upregulated in Lung Cancer and Promotes Cell Progression and Proliferation

Firstly, we evaluated the HOTAIR level from four LC cell lines and health MCF-10A cells with qRT-PCR. HOTAIR in LC cells were greatly upregulated than normal (Figure 1(a)). We created HOTAIR-depleted LC cells based on the spontaneous transcriptional level of HOTAIR in LC cells (Figure 1(b)). The CCK-8 experiment revealed that removing HOTAIR significantly reduced tumor growth in LC cells (Figures 1(c) and 1(d)). To determine the impact of HOTAIR transcription on cell viability, flow cytometry was used to examine apoptotic death in LC pretreated with or without si-HOTAIR for 48 hours. In comparison to si-NC cells, HOTAIR-depleted LC cells exhibited greater apoptosis (Figure 1(e)). The impact of lncRNA HOTAIR transcription on cell growth was also investigated. When compared with the si-NC groups, the proportion of EdU-positive cells was considerably lower in HOTAIR-depleted clusters (Figure 1(f)). In LC cells, lncRNA HOTAIR depletion improved ADR sensitivities, increased cell apoptosis and DNA damage, and limited cell proliferation, according to these findings.

### 3.2. HOTAIR Knockdown Dampens the Aerobic Glycolysis in LC Cells

Considering the relationship of aerobic glycolysis and tumor progression, HOTAIR was tested in LC cells to see if it influenced glycolysis. Initially, HOTAIR knockdown of LC cells markedly reduced glucose acquisition (Figure 2(a)), lactic generation (Figure 2(b)), and ATP generation (Figure 2(c)). In addition, HOTAIR depletion in LC cells resulted in a lower external acidity ratio (ECAR), which is a measure of cellular total glycolysis flow (Figures 2(d) and 2(e)). Moreover, oxygen consumption rate (OCR), an indicator of mitochondrial respiration, was significantly increased in HOTAIR knockdown LC cells (Figures 2(f) and 2(g)). These findings strongly recommended that HOTAIR was implicated in the control of glycolytic pathway in LC cells.

### 3.3. HOTAIR Associates with HK2 mRNA and Promotes Its Stability

We extracted RNA and then measured HOTAIR transcription to investigate the addressing principle of HOTAIR in LC cells. HOTAIR was mostly located in the cellular plasm (Figure 3(a)), implying that it is involved in posttranscriptional control. We used MS2-binding protein (MS2bp), which specifically binds RNA with MS2-binding motifs, in a RIP test (MS2bs). LC cells were found with a vector producing MS2bp-GFP after a vector amount of power HOTAIR coupled with MS2bs components was generated. The GFP reagent was then used to conduct the RIP. The mRNA trapped by HOTAIR was then analyzed using PCR. The restricting component of glucose, HK2, was one of the most abundant transcripts, which was surprising. We used a RIP experiment to confirm HOTAIR's direct contact with HK2 mRNA, and the results showed that the HOTAIR RIP in LC cells was considerably preferential for HK2 mRNA when comparing to the blank vectors or IgG (Figure 3(b)). The interaction between HOTAIR and HK2 mRNA was then validated by the results of an RNA knock test (Figure 3(c)).

The regulating link of HOTAIR and HK2 was then identified. In LC cells, knocking down HOTAIR resulted in a substantial reduction in HK2 mRNA and protein expression (Figures 3(d) and 3(e)). We produced transient expression plasmids well with HK2 regulatory regions and transfected it into LC cells with the HOTAIR change. HOTAIR reduction, on the other hand, had no effect on the fluorescence activation of the HK2 regulator, implying HOTAIR controlled HK2 output through a posttranscriptional mechanism (Figure 3(f)). Seeing if HOTAIR influenced HK2 mRNA breakdown, LC cell with HOTAIR mutations was incubated with the RNA biosynthesis blocker and the disappearance of HK2 mRNA was assessed. HOTAIR knockdown reduced the 50% life of HK2 mRNA in LC cells (Figure 3(g)). Our data show that HOTAIR increased HK2 transcription via increasing the reliability of HK2 mRNA.

### 3.4. HOTAIR Upregulates HK2 Expression via Association with RNA De-methyltransferase FTO

N6-methyladenosine (m6A) alteration was discovered recently to regulate quickly realized RNA durability. As a result, we investigated the role of m6A alteration in the HOTAIR-mediated control of HK2 downregulation. We performed a MeRIP experiment and discovered that m6A antibody significantly enriched HK2 mRNA relative to IgG (Figure 4(a)). Furthermore, HOTAIR depletion significantly elevated m6A methylation of HK2 mRNA in LC cells (Figure 4(b)). These findings suggested that HOTAIR could inhibit the m6A alteration of HK2 mRNA.

FTO and ALKBH5 both function as m6A de-methyl erases. Then, we look into which m6A de-methyl erase FTO and ALKBH5 were involved in HOTAIR-mediated PTEN m6A transformation. FTO and ALKBH5 antibodies were used in a RIP assay. The findings demonstrated that FTO antibody, rather than ALKBH5, may considerably enhance HOTAIR proteins (Figure 4(c)). To add to the evidence, knocking down HOTAIR dramatically reduced FTO bound in HK2 mRNA (Figure 4(d)). Furthermore, FTO upregulation prevented si-HOTAIR-induced HK2 downregulation and degradation (Figure 4(e)). Our findings revealed that HOTAIR, through its interaction with FTO, favorably controlled m6A alteration of HK2 mRNA.

### 3.5. HOTAIR/FTO/HK2 Axis Facilitates LC Proliferation and Proliferation

Recovery studies were conducted to verify the involvement of the HOTAIR/FTO/HK2 axis in LC growth. First, Western blot results showed that HOTAIR removal decreased HK2 expression levels, while HK2 amplification could partly restore HK2 expression (Figure 5(a)). Furthermore, HK2 amplification could partially repair HOTAIR knockdown's tumor suppressor effect in LC cells (Figures 5(b) and 5(c)). These findings suggested that the HOTAIR/Fto/Hk2 axis boosted cell growth and development in LC cells via modulating gluconeogenesis.

## 4. Discussion

Chemotherapy is one of the most important treatment approaches for lung cancer patients. Nevertheless, pulmonary chemotherapy continues to be hampered by growth. The detailed mechanisms of LC proliferation are important for improving the efficiency of chemotherapy. Therefore, we would like to know a proliferation biomarker and the pathways addressing development of proliferation of LC. We further discovered that sevoflurane decreased the expression of lncRNA HOTAIR and attenuated the proliferation of LC in vitro.

Increasing data suggests that lncRNAs serve critical functions in a variety of malignant physiological systems, like proliferation and migration; lncRNA ANCR increases tumorigenesis and growth in carcinoma through suppressing PTEN [17]. In female tumors, upregulation of HOTAIR causes proliferation via promoting HIF-1*α* expression [18]. Recently, a novel conserved lncRNA “HOX Transcript Antisense RNA” (HOTAIR) has been characterized, and some researches had believed HOTAIR was increased in stomach tumor, colorectal cancer, and hepatocellular carcinoma and played pivotal roles in cancer regulation [19, 20]. Recently, HOTAIR has been found to promote drug-resistant strains and malignancy cell growth. Nevertheless, the functions and molecular networks of HOTAIR in LC remain uncertain. We observed HOTAIR induced in LC. Functionally, the knockdowned HOTAIR repressed cellular growth and resisted to chemotherapy. Moreover, we demonstrated that HOTAIR promotes LC growth and proliferation in a m6A dependency mode. Thus, our study firstly showed that HOTAIR promotes LC development and proliferation.

This one has been observed that lncRNAs can bind to RBPs and improve the stability of target mRNAs [21]. CASC9, for example, increases TGF-mRNA stabilization by connection with CPSF3, promoting tumorigenesis and dissemination in colon cancer [22]. LINC01093 easily connects to IGF2BP1 and disrupts its connection with carcinogen GLI1 mRNA, causing GLI1 mRNA breakdown and inhibiting HCC cell growth and dissemination [23]. lncRNA-Assisted Stability of Transcripts (LAST) has been found to improve CCND1 mRNA stable by collaborating with CNBP to attach to the CCND1 mRNA 5 0 UTR [24]. HOTAIR was validated to straightly enhance HK2 expression and mRNA stabilization. These findings provided sufficient proof that HOTAIR promoted LC proliferation by directly stabilizing HK2 mRNA.

Cancerous cells have an abnormal metabolism due to strong glycolytic pathway (referred as the Warburg effect), an elevated blood glucose absorption rates, and rapid lactate generation [10, 25]. Emerging evidence demonstrated that the elevated aerobic glycolysis in malignancies strongly correlates to proliferation owing to upregulating the endogenous antioxidant capacity through the addition of glucose and lactic; the anaerobic glycol cycle could be used to treat cancer [9, 26, 27]. However, whether lncRNAs play a role in glycolytic pathway and proliferation in LC remain unclear. Previously, 3-phosphoinositide-dependent protein kinase 1 (HK2) is upregulated in several kinds of carcinomas and associated with worse prognosis [28]. A recent study indicated that targeted HK2 with DAP inhibited AML cell growth via multiple signaling pathways and suggest that targeting HK2 may be promising therapy strategies for AML [29]. Nevertheless, the upstream regulation mechanism of HK2 and function in proliferation in LC remain unclear. In the present study, HOTAIR knockdown could inhibit HK2 expression and aerobic glycolysis process via the reeducations of glucose metabolism, lactate generation, ATP generation, and ECAR, demonstrating the important role of HK2 in aerobic glycolysis and proliferation in LC. Importantly, HOTAIR regulates the FTO/HK2 pathway and regulates glycogen synthesis, according to me-RIP tests and rescuing investigations. It was the first time the HOTAIR/FTO/HK2 circuit has been discovered, and it presents a feasible route for potential treatment drugs that target glycogen synthesis in LC. Lately, RNA epigenetics became a fascinating subject of medical research. In humans' malignant illnesses, the m6A alteration is among the most prevalent and essential mRNA changes [14, 30]. An increasing data suggests that m6A's “writers,” “erasers,” and “readers” play a key role in carcinoma beginning and progression. FTO was discovered to be one of the first “erasers” of m6A, and it has been linked both to enhanced body fat and overweight, as well as the advancement of many cancers [31]. The abundance and effects in cancer of m6A on RNA are determined by the dynamic interplay between its methyltransferases (“writers”), binding proteins (“readers”), and demethylases (“erasers”). Originally, the correlation between FTO single-nucleotide polymorphisms or overweight and the likelihood of malignancy beginning was heavily focused on throat, mammary, prostate, renal, pancreas, and endometrium cancers [32]. Nonetheless, FTO's carcinogenic role in mRNA epigenetic modification was just discovered [30]. FTO transcription was discovered to be high in AML, and knocking down FTO within those peripheral blood lymphocytes resulted in an antitumor profile. FTO has been demonstrated to alter the stability of ASB2 and RARA transcripts by demethylating mRNA [33]. The carcinogenic role of FTO was discovered via mRNA epigenetic modification in this research, suggesting that inhibiting FTO could be a potent anticancer therapeutic approach [33]. In our study, we found that HOTAIR promoted the stabilization of HK2 in a FTO dependency mode in lung cancer. The findings of this research confirmed FTO's carcinogenic involvement in malignancy, as well as the link with FTO-modulated mRNA epigenetic modification and LC treatment tolerance. The same idea can be found in the study put forward by Liang et al. [34]. They have applied new methods in the study, and the conclusions drawn can also give some support to this study.

In conclusion, we established that the HOTAIR/FTO/HK2 loop can affect the susceptibility of LC cells to chemo treatments by regulating glycogen synthesis. Our results add to our understanding of LC multiplication and suggest that using HIFU to address the HOTAIR/FTO/HK2 pathway could be a potential technique for improving the effectiveness of LC treatment. In the future, we will deeply study how HOTAIR is coupled with hexokinase 2 (HK2) mRNA and affects HK2-mediated LC. In addition, we will further study the specific mechanism of HOTAIR affecting LC glycogen through HK2.

## Figures and Tables

**Figure 1:** HOTAIR is activated, allowing cells to grow and proliferate. (a) Assessment of HOTAIR transcription using qRT-PCR in 4 distinct LC cell lines and healthy cells. (b) HOTAIR transcription in LC cells were transfected with either a negative control shRNA (si-NC) or a HOTAIR shRNA (si-HOTAIR). (c and d) The CCK-8 test was used to identify cell growth in standard and HOTAIR-depleted LC cells. (e) Annexin-V FITC techniques were used to determine the apoptotic rate in normal and HOTAIR-depleted LC cells. (f) EDU testing methods used to determine the EDU higher accuracy of normal and HOTAIR-depleted LC cells. ^∗^*P* 0.05 when compared to the control.

**Figure 2:** HOTAIR depletion reduces glycogen synthesis in LC cells. (a) The glucose uptake of LC cell was measured. (b) LC cell lactic generation was assessed. (c) The ATP of LC cell was evaluated. (d and e) The extracellular acidification rate (ECAR) of LC cell was measured using a Seahorse Bioscience XFp analyzer. (f and g) The O_2_ intake (OCR) of LC cell was measured using a Seahorse Bioscience XFp analyzer. Findings are given as mean SD. ^∗^*P* 0.05 when opposed to the negative control.

**Figure 3:** HOTAIR binds to HK2 mRNA and enhances its stabilization. (a) The localization of HOTAIR in LC cell was evaluated by subcellular fractionation and qRT-PCR. (b) MS2-RIP and qRT-PCR were used to detect HK2 mRNA related with HOTAIR in LC3 cell. (c) Biotin-labeled HOTAIR was treated with LC lysates. qRT-PCR was used to assess the level of HK2 mRNA in the knock condition. (d) Western blot examination of HK2 transcription in HOTAIR-depleted LC cell and normal cells. (e) qRT-PCR study of HK2 transcription in HOTAIR-depleted LC cell and standard cells. (f) Standard and HOTAIR-depleted LC cells were infected with a luciferase plasmid containing nothing or the HK2 promoter region. The luciferase activity was evaluated after 48 hours. (g) A-amanitin (50 mM) was used to prevent fresh RNA production in standard and HOTAIR-depleted LC cells. The quantities of HK2 mRNA were identified at the specified time points. ^∗^*P* value more than 0.05 compared to the controls.

**Figure 4:** HOTAIR upregulates HK2 expression via association with RNA de-methyltransferase FTO. (a) MeRIP assay was used to detect the m6A modification of HK2 mRNA in LC cells. (b) MeRIP assay was used to detect the m6A modification of HK2 mRNA in control and HOTAIR-depleted cells. (c) RIP assay using IgG, FTO, or ALKBH5 antibody was performed in LC cells. The pull-down HOTAIR was then detected using qRT-PCR. (d) The RIP assay using IgG or FTO antibody was performed in control and HOTAIR-depleted LC cells. (e) Overexpression of FTO recued the degradation of HK2 mRNA mediated by HOTAIR knockdown. ^∗^*P* < 0.05 compared with the negative control.

**Figure 5:** The HOTAIR/FTO/HK2 axis promotes LC proliferation and growth. (a) The activation of the HK2 protein in LC cells was discovered using a Western blot experiment. (b and c) On the CCK8 test of LC cells, HK2 amplification partially restored the inhibitory effects of HOTAIR depletion. The data is presented as a mean standard deviation. ^∗^*P* 0.05 when compared to the negative control group. When compared to the si-HOTAIR group, ^#^*P* 0.05.

## Data Availability

The data that support the findings of this study are available from third-party rights, but restrictions apply to the availability of these data, which were used under license for the current study, and so are not publicly available.

## Additional Points

*Highlights*. (1) HOTAIR was upregulated in lung cancer. (2) Sevoflurane induced knockdown of HOTAIR of lung cancer cells by inhibition of aerobic glycolysis. (3) Our study firstly demonstrated a m6A-dependent regulatory mechanism among HOTAIR, FTO, and HK2 existed in lung cancer. (4) The HOTAIR/FTO/HK2 axis regulated the aerobic glycolysis and proliferation of lung cancer.
